The article "Effect of Resveratrol Combined with Donepezil Hydrochloride on Inflammatory Factor Level and Cognitive Function Level of Patients with Alzheimer's Disease" was retracted in 2023. Reason: concerns about the peer review.

# Effect of Resveratrol Combined with Donepezil Hydrochloride on Inflammatory Factor Level and Cognitive Function Level of Patients with Alzheimer's Disease

**DOI:** 10.1155/2022/9148650

**Published:** 2022-03-25

**Authors:** Xincui Fang, Jing Zhang, Jianping Zhao, Litao Wang

**Affiliations:** ^1^The Psychological Hospital, Qingdao Mental Health Center, Qingdao 266034, Shandong Province, China; ^2^The Seventh Psychiatry Ward, Qingdao Mental Health Center, Qingdao 266034, Shandong Province, China; ^3^Qingdao University, 308 Ningxia Road, Qingdao 266071, Shandong Province, China

## Abstract

**Objective:**

To explore the effect of resveratrol (RES) combined with donepezil hydrochloride on inflammatory factor level and cognitive function level of patients with Alzheimer's disease (AD).

**Methods:**

A total of 90 AD patients treated in our hospital from June 2019 to June 2020 were selected as the study objects and divided into the control group (CG) and experimental group (EG) by the randomized and double-blind method, with 45 cases each. Patients in CG received donepezil hydrochloride treatment, and on this basis, those in EG received additional RES treatment, so as to compare the clinical indicators between the two groups.

**Results:**

Compared with CG after treatment, EG obtained significantly higher good rate, MMSE score, and FIM score (*P* < 0.05) and obviously lower clinical indicators and ADAS-cog score (*P* < 0.001), and between CG and EG, no obvious difference in total incidence rate of adverse reactions was observed after treatment (*P* > 0.05).

**Conclusion:**

Combining RES with donepezil hydrochloride has significant clinical efficacy in treating AD, which can effectively improve patients' inflammatory factor indicators, promote their cognitive function, and facilitate patient prognosis.

## 1. Introduction

Alzheimer's disease (AD), also known as senile dementia, is one of the 4th leading causes of death after stroke, heart disease, and cancer. The pathogenesis of AD is still unclear, and some scholars suggest that it may be due to restricted interests, heredity, psychological stress, and eccentric personality. In addition, age, positive family history, Down's syndrome, mild cognitive impairment, chronic diseases, low education level, and less social activities are all risk factors triggering AD. Relevant data show that AD patients aged 60–65 years account for less than 1%, and the incidence increases in the population aged over 65 years [1]. It has been reported that the proportion of AD patients over 85 years old is 25%–32% in western countries [2]. Data from the *World Alzheimer Report 2016* released by Alzheimer's Disease International (ADI) indicate that there are approximately 9.5 million patients with dementia in China, accounting for 20% of the global total [3]. By 2030, the number of patients with dementia in China will likely exceed 16 million. Currently, over 5 million people throughout the United States are deeply afflicted with AD, and every 65 seconds, there will be 1 new AD case in the United States, and hence the number of AD patients will likely approach 16 million by 2050 [4]. In addition, AD is also the sixth leading cause of death in the United States. With the increasing pace of social aging, AD has gradually become a considerable social problem.

As a neurodegenerative disease, AD is a brain disorder characterized by a general loss of neurological abilities such as memory, judgment, language, and abstract thinking. The course of the disease is usually divided into early (memory impairment, visual-spatial disorientation, etc.), middle (loss of independent living ability), and late (severe mental decline, limb rigidity, etc.), and finally, most patients die from accompanying infections. At present, there is no specific medicine to cure AD or reverse the course of AD, but combined drug therapy is able to delay the progression of the condition and alleviate the clinical symptoms. Resveratrol (RES) was first discovered in 1940 and subsequently proven to have therapeutic effects against cardiovascular diseases [5]. Osborn et al. [6] pointed out that RES has immune regulation and neuroprotective effects. In recent years, this drug has gained increasing attention in the treatment of neurodegenerative diseases. Donepezil hydrochloride is widely used in the clinical treatment of AD with definite efficacy and is one of the first drugs approved by the US Food and Drug Administration (FDA) for the treatment of AD [7]. In addition, controlled studies have suggested that the single use of the two drugs has beneficial effects on cognitive dysfunction and psychotic symptoms, but the effects of their combination have rarely been reported [8]. Based on this, the combined therapy was adopted herein to observe its effect on inflammatory factor level and cognitive function level of patients after treatment, so as to analyze the application value of such treatment scheme.

## 2. Materials and Methods

### 2.1. General Data

A total of 90 AD patients treated in our hospital from June 2019 to June 2020 were selected as the study objects and divided into the control group (CG) and experimental group (EG) by the randomized and double-blind method, with 45 cases each.

### 2.2. Enrollment of Study Objects

Inclusion criteria were as follows: ① the patients met the diagnostic criteria for AD in the *Diagnostic and Statistical Manual of Mental Disorders* (DSM-V) [9]; ② the patients had to be sent to the psychiatric ward and required hospitalization due to aggressive, psychiatric, or agitated signs and symptoms so severe that could damage self-cognitive function, and treatment with anti-psychotics was considered reasonable by the clinician; ③ 7 d before registration, the patients' psychiatric or slightly agitated symptoms happened daily; ④ the patients were hospitalized during the study; ⑤ the patients had complete clinical data; and ⑥ the study met the World Medical Association Declaration of Helsinki [10].

Exclusion criteria for patients were as follows: ① complicated with other nervous system diseases and organ dysfunction; ② drug allergy; ③ complicated with malignant tumors or suspected malignant lesions; ④ complicated with abnormal immune function, infectious diseases, and endocrine dysfunction; ⑤ drug abuse; ⑥ suffering from delirium or primary mental disorder (e.g., schizophrenia); and ⑦ participating in other drug trails.

## 3. Methods

### 3.1. Routine Intervention

Before the study started, patients in the two groups received physical examination and safety measurement, with the indicators including routine blood test, creatinine, alanine aminotransferase (ALT), and total bilirubin level, and the results were within the normal range.

#### 3.1.1. CG

Initially, patients in CG orally took 5 mg of donepezil hydrochloride (manufacturer: Shaanxi Ark Pharmaceutical Co. Ltd.; NMPA approval no. H20030583; specification: 5 mg *∗* 7 s) once daily before sleep, and after taking the drug for more than 1 month, the dosage could be adjusted to 10 mg once daily according to the treatment effect.

#### 3.1.2. EG

On this basis, patients in EG took 1 or 2 RES tablets (manufacturer: Jining Hengkang Biotechnology Co. Ltd.; China health food approval no. G20130044; specification: 1.0 g *∗* 60 tablets) daily as dietary supplement. The administration, time, and dosage of donepezil hydrochloride were the same as those in CG. Patients in the two groups were treated for 2 months.

### 3.2. Observation Indicators

The good rate of treatment effect was compared between the two groups. It was regarded as excellent if patients' symptoms such as memory decline and poor mental status were obviously alleviated, the MMSE score was more than 5 points, and patients could take care of themselves; it was regarded as good if patients' symptoms such as memory decline and poor mental status were alleviated, the MMSE score was 1–4 points, and patients could take care of themselves to some extent; and it was regarded as poor if patients failed to meet the aforesaid standards. Good rate = (number of excellent cases + number of good cases)/total number of cases *∗* 100%.

Five milliliter of fasting venous blood was drawn from the patients in the two groups in the morning, the serum was separated after centrifugation, and the supernatant was extracted. All serum specimens were placed under −80°C, and the serum interleukin-6 (IL-6) and tumor necrosis factor *α* (TNF-*α*) in the specimens were measured in strict accordance with the specification on ELISA kits (manufacturer: Shanghai Tongwei Industry Co. Ltd.). At the same time, patients' midstream urine in the morning was reserved for measurement of Alzheimer-associated neuronal thread protein (AD7c-NTP) indicator by enzyme-linked immunosorbent assay (ELISA), and all operations were conducted strictly according to the specification on the kits (manufacturer: BOSK Bio, Wuhan).

The cognitive function after treatment of patients in the two groups was assessed by referring to Mini-Mental State Examination (MMSE) [11] and Alzheimer's Disease Assessment Scale-Cognitive Subscale (ADAS-cog) [12]. The MMSE scale contained orientation (10 points), memory (3 points), attention and calculation (5 points), recall (3 points), and language (9 points), and the total score was 30 points, with lower scores indicating more serious dementia (27–30 points indicated normal, and <27 points indicated cognitive impairment). The severity of dementia was graded by MMSE as follows: ≥21 points indicated mild dementia, 10–20 points indicated moderate dementia, and ≤9 points indicated severe dementia. The ADAS-cog scale consisted of 12 items, including naming objects and fingers, word recall, ideational praxis, word recognition, execution of verbal command, language, remembering test instructions, word finding difficulty, comprehension of spoken language and exercises on attention, orientation, structure, and intention, which were used to assess the most important cognitive impairment in AD, including domains of memory, language, operational ability, and attention. The total score of ADAS-cog was 75 points, with higher scores indicating more serious cognitive impairment.

The daily living ability after treatment of patients in the two groups was evaluated by Functional Independence Measure (FIM) [13], which included mobility (self-care ability, sphincter control, transfer, walking, etc.), and cognitive function (communication and social cognition). The maximum score was 126 points (91 points for mobility and 35 points for cognitive function), and the minimum score was 18 points, with higher scores indicating better daily living ability.

Follow-up was performed to patients by means of telephone, WeChat, interview, etc., once every 2 weeks, and 4 times in total, so as to record the incidence rates of limb weakness, dizziness, nausea, and diarrhea of patients during treatment.

### 3.3. Statistical Processing

In this study, the data processing software was SPSS20.0, the picture drawing software was GraphPad Prism 7 (GraphPad Software, San Diego, USA), the items included were enumeration data and measurement data, the methods used were *X*^2^ test, *t*-test, and normality test, and differences were considered statistically significant at *P* < 0.05.

## 4. Results

### 4.1. Between-Group Comparison of Baseline Data

No significant differences in gender, mean age, BMI value, mean duration of disease, educational degree, religious faith, occupation, personal monthly income, smoking, drinking, and place of residence between the two groups were observed (*P* > 0.05) (see Table 1).

### 4.2. Between-Group Comparison of Good Rate

The good rate was obviously higher in EG than in CG (*P* < 0.05) (see Table 2).

### 4.3. Between-Group Comparison of Clinical Indicators after Treatment

After treatment, various clinical indicators were obviously lower in EG than in CG (*P* < 0.001) (see Table 3).

### 4.4. Between-Group Comparison of MMSE and ADAS-Cog Scores after Treatment

Compared with CG after treatment, EG obtained obviously higher MMSE score (*P* < 0.001) and significantly lower ADAS-cog score (*P* < 0.001) (see Figure 1).

### 4.5. Between-Group Comparison of FIM Score after Treatment

Compared with CG after treatment, EG obtained obviously higher FIM score (*P* < 0.001) (see Figure 2).

### 4.6. Between-Group Comparison of Adverse Reaction Rate

Although no obvious difference in total incidence rate of adverse reactions between EG and CG after treatment was observed (*P* > 0.05), the number of cases with adverse reactions was lower in EG than in CG (see Table 4).

## 5. Discussion

The main symptom of AD patients is progressive decline in cognitive function, and some patients also present a variety of violent, agitating, and yelling behaviors, which lead to many adverse effects for clinical treatment and care. Jin et al. [14] indicated that about 55% of AD patients in clinic would develop dementia with persistent confusion and anxiety. With the increasing aging trend, AD has gradually become a major cause affecting the physical health of the elderly population [15]. Some scholars believe that the occurrence of AD is related to the damage of the central cholinergic nervous system in the brain, so acetylcholinesterase inhibitor (AChEI) plays a key role in treatment. Donepezil hydrochloride, a second-generation reversible AChEI developed by Eisai Pharmaceutical Company in Japan in the late 1980s, which was approved by the US FDA in 1996 and became available in the US in 1997, is currently available in more than 40 countries and regions worldwide [16]. This drug is a reversible, highly selective, and long-acting AChEI, which primarily inhibits acetylcholinesterase activity in the brain with its specificity, thereby increasing the concentration of acetylcholine, overcoming problems such as memory decline triggered by choline deficiency, and further improving cognitive function in AD patients [17, 18]. However, some patients did not achieve satisfactory outcomes with donepezil hydrochloride alone. For example, anti-oxidant drugs need to be administered to patients in the early stage of disease, but it is difficult to achieve the expected anti-oxidant effect alone, and nonsteroidal anti-inflammatory drugs only play a protective role during administration, and the single application cannot reverse the course of pathological deterioration in AD patients. The study by Xu et al. [19] showed that the overall efficiency of donepezil hydrochloride alone was 68.50%. In this study, the good rate of EG was significantly higher than that of CG (*P* < 0.05), indicating that drug combination was more effective than single drug administration. As a multifunctional cytokine, IL-6 can affect antigen-specific responses, participate in inflammation, and regulate the responses in the acute phase, which is very important in the immune system. TNF-*α* is a cytokine implicated in systemic inflammation that also belongs to a group of numerous cytokines causing acute phase responses, and it is related to a number of human diseases, including AD. AD7c-NTP, a neuronal thread protein mediated in neurons and localized to axons undergoing neurogenesis, is elevated in the cerebrospinal fluid and urine of AD patients and positively correlates with the severity of dementia. Compared with CG after treatment, EG obtained obviously lower clinical indicators (*P* < 0.001), demonstrating that drug combination could effectively inhibit the expression of inflammatory factors and improve patients' clinical indicators. The reason for such results was that resveratrol showed good therapeutic effects against AD in vitro, and its retarding effect on AD was manifested in the interference of amyloid-*β* peptide (A*β*) formation, stabilization of the relative protein action of microtubules, inhibition of inflammatory response, and improvement of anti-oxidant effect, thereby exerting neuroprotective effects [20]. Liu et al. [21] indicated that RES, a polyphenolic compound with neuroprotective properties, plays a role in oxidation resistance, anti-inflammation, anti-cancer, and anti-amyloid protein and can resist AD in in vivo and in vitro tests. RES is a non-flavonoid polyphenolic compound extracted from a variety of fruits, and its therapeutic potential has been widely applied due to its diverse properties [22]. Relevant studies have reported that RES has shown significant clinical efficacy in in vitro models of Parkinson's disease, AD, epilepsy, amyotrophic lateral sclerosis, Huntington's disease, and neurological impairment [23, 24]. The study by De Carli et al. [25] analyzed and elucidated the key signaling pathways and molecular mechanisms of KEGHG pathway and found that RES could improve cognitive function in AD patients through ADA*β* and tau pathological process. The study results showed that the MMSE score and ADAS-cog score were obviously better in EG than in CG after treatment (*P* < 0.001), indicating that combining RES with donepezil hydrochloride could improve the cognitive function, self-care ability, and functional independence of AD patients. Moreover, the FIM score was obviously higher in EG than in CG after treatment (*P* < 0.001), demonstrating that drug combination could enhance the treatment effect, which may be related to the protective mechanism of RES and donepezil hydrochloride on multiple targets and links in the central nervous system. Also, the study found no obvious difference in the total incidence rate of adverse reactions between the two groups, proving that the combination was safe and reliable in treating AD. There are certain limitations in this study. First, the study was based on the population within our region and did not include a sufficient number of patients from other provinces and other ethnic groups, so the results may be affected by small sample size, geographical culture, and ethnic differences, and further refined experimental design is necessary; second, long-term follow-up observation of the intervention effect of patients was lacking; finally, scales were still the method for clinical evaluation, so there must be certain subjective and intentions when patients were answering the questions, which might affect the final results of the clinical trial to some extent. So, the long-term safety and efficacy will be evaluated by close follow-up in the future. Also, well-designed prospective studies are required to obtain higher-grade evidence as a reference basis for AD treatment, so as to benefit more patients. To sum up, the conclusion obtained initially in this study remains to be refined by more subsequent studies.

## Figures and Tables

**Figure 1:** Between-group comparison of MMSE and ADAS-cog scores after treatment ($\bar{\text{x}}$ ±*s*). (a) showed the between-group comparison of MMSE score after treatment, the horizontal axis indicated EG and CG, and the vertical axis indicated the MMSE score (points); the MMSE scores of EG and CG were, respectively, (22.00 ± 1.60) and (17.07 ± 1.47), and ∗ indicated obvious between-group difference in MMSE scores after treatment (*t* = 15.221, *P* < 0.001). (b) showed the between-group comparison of ADAS-cog score after treatment, the horizontal axis indicated EG and CG, and the vertical axis indicated the ADAS-cog score (points); the ADAS-cog scores of EG and CG were, respectively, (18.04 ± 2.06) and (22.02 ± 2.55), and ∗∗ indicated obvious between-group difference in ADAS-cog scores after treatment (*t* = 8.144, *P* < 0.001).

**Figure 2:** Between-group comparison in FIM score after treatment ($\bar{\text{x}}$ ± *s*). The horizontal axis indicated EG and CG, and the vertical axis indicated the FIM score (points); the mean FIM scores of EG and CG after treatment were, respectively, (93.80 ± 2.55) and (85.13 ± 2.96), and ∗ indicated significant between-group difference in mean FIM scores after treatment (*t* = 14.886, *P* < 0.001).

**Table 1:** Between-group comparison of baseline data.

Item	EG (*n* = 45)	CG (*n* = 45)	*x* ^2^/*t*	*P*
Gender			0.046	0.830
Male	27 (60.00%)	26 (57.78%)		
Female	18 (40.00%)	19 (42.22%)		
Mean age ($\bar{\text{x}}$ ± *s*, years)	69.22 ± 4.67	69.47 ± 3.96	0.274	0.785
BMI (kg/m^2^)	20.15 ± 0.51	20.06 ± 0.26	1.055	0.295
Mean duration of illness ($\bar{\text{x}}$ ± *s*, years)	2.02 ± 0.84	2.33 ± 1.15		
Educational degree				
Primary school and junior high school	15 (33.33%)	14 (31.11%)	0.051	0.822
Senior high school and junior college	14 (31.11%)	16 (35.56%)	0.200	0.655
College and above	16 (35.56%)	15 (33.33%)	0.049	0.824
Religious faith			0.051	0.822
Yes	15 (33.33%)	14 (31.11%)		
No	30 (66.67%)	31 (68.89%)		
Occupation				
Farmer	5 (11.11%)	6 (13.33%)	0.104	0.748
Worker	4 (8.89%)	5 (11.11%)	0.124	0.725
Teacher and civil servant	18 (40.00%)	17 (37.78%)	0.047	0.829
Retired	14 (31.11%)	13 (28.89%)	0.053	0.818
Others	4 (8.89%)	4 (8.89%)	0.000	1.000
Personal monthly income (yuan)				
<2000	4 (8.89%)	5 (11.11%)	0.124	0.725
2000–5000	20 (44.44%)	21 (46.67%)	0.045	0.832
5000–8000	21 (46.67%)	19 (42.22%)	0.180	0.671
Smoking			0.045	0.832
Yes	21 (46.67%)	20 (44.44%)		
No	24 (53.33%)	25 (55.56%)		
Drinking			0.045	0.833
Yes	23 (51.11%)	24 (53.33%)		
No	22 (48.89%)	21 (46.67%)		
Place of residence			0.047	0.829
Urban area	27 (60.00%)	28 (62.22%)		
Rural area	18 (40.00%)	17 (37.78%)		

**Table 2:** Between-group comparison of good rate (*n* (%)).

Group	*n*	Excellent	Good	Poor	Good rate
EG	45	25 (55.56%)	18 (40.00%)	2 (4.44%)	43 (95.56%)
CG	45	17 (37.78%)	16 (35.56%)	12 (26.67%)	33 (73.33%)
*x* ^2^					8.459
*P*					<0.05

**Table 3:** Between-group comparison of clinical indicators after treatment ($\bar{\text{x}}$ ±  *s*).

Group	*n*	IL-6 (ng/L)	TNF-*α* (ng/L)	AD7C-NTP (ng/mL)
EG	45	60.48 ± 12.09	143.93 ± 9.72	6.92 ± 0.57
CG	45	121.71 ± 16.83	172.71 ± 13.80	9.00 ± 0.56
*T*		19.821	11.438	17.462
*P*		<0.001	<0.001	<0.001

**Table 4:** Between-group comparison of adverse reaction rate (*n* (%)).

Group	*n*	Dizziness	Limb weakness	Nausea	Diarrhea	Total incidence rate
EG	45	1 (2.22%)	0 (0.00%)	1 (2.22%)	0 (0.00%)	2 (4.44%)
CG	45	2 (4.44%)	1 (2.22%)	2 (4.44%)	1 (2.22%)	6 (13.33%)
*x* ^2^						2.195
*P*						0.138

## Data Availability

The data used to support the findings of this study are available on reasonable request from the corresponding author.
